The article "Application of a Computerized Decision Support System to Develop Care Strategies for Elderly Hemodialysis Patients" was published in 2021. Journal: J Healthc Eng.

# Application of a Computerized Decision Support System to Develop Care Strategies for Elderly Hemodialysis Patients

**DOI:** 10.1155/2021/5060484

**Published:** 2021-06-19

**Authors:** Yiqiu Zhu, Xiyi Zheng

**Affiliations:** The First Affiliated Hospital of Soochow University, Suzhou 215000, Jiangsu, China

## Abstract

In this paper, the strategy of elderly haemodialysis patients' care is analysed by the computer's decision system to conduct an in-depth research machine. Maintenance haemodialysis patients have a high demand for continuation care, and healthcare workers should provide personalized and specialized seamless continuation care services for patients according to patients' needs, by reasonably using the hospital, community, and other health resources and with the help of emerging network technologies, such as information platforms and wearable devices to prolong the survival period of patients and improve their self-management ability and quality of life. The service provision and compensation strategy of the combined healthcare model should be optimized to improve the health protection of the elderly and promote health equity. On the one hand, it should target strengthening the service provision of healthcare integration, guide the elderly to reasonably choose the healthcare integration model, and pay attention to the spiritual and cultural needs and end-of-life care services for the elderly. On the other hand, we should expand the financing channels of medical insurance, optimize the design of compensation mechanisms, explore the role of health risk sharing, and accelerate the development of long-term care insurance, independent of basic medical insurance. The reliability of the scale was found to be 0.916 for the total Cronbach alpha coefficient, 0.798–0.919 for each dimension, and 0.813 for the fold-half reliability of the scale; the validity indicated that the correlation coefficient range of each article day with the total scale score was 0.27–0.72, and the correlation coefficient range of each dimension with the total scale was 0.56–0.72. The validation factor analysis was used to verify the structure of the scale. The validation factor analysis indexes met the fitting criteria after correction. The model fitted better with the actual model after correction, indicating that the scale has good reliability.

## 1. Introduction

End-stage renal disease (ESRD) is the final stage of various chronic kidney diseases when patients have irreversible impairment of kidney function and need to rely on kidney transplantation or dialysis therapy to maintain their lives [1]. Given the limited number of kidney donors and the high cost of transplantation, most ESRD patients can only choose dialysis therapy. The current dialysis therapies include hemodialysis (HD) and peritoneal dialysis (PD). MHD patients' survival and quality of life are often compromised by the irreversible disease process, complications, specificity of the haemodialysis treatment modality and treatment environment, and water and activity restrictions [2]. Most patients return to their homes, and due to the lack of guidance and supervision by healthcare professionals, their self-management will be lax, making it difficult to adhere to long-term self-monitoring, diet, and water control, which in turn affects the effectiveness of dialysis, increases the risk of complications and adverse outcomes, and increases the burden on families and society.

The article "Application of a Computerized Decision Support System to Develop Care Strategies for Elderly Hemodialysis Patients" was published in 2021. Journal: J Healthc Eng.

Patients on long-term dialysis are prone to malnutrition due to disease consumption, dietary restrictions, and treatment effects, and related studies have shown that the incidence of malnutrition in haemodialysis patients ranges from 37.50% to 86.0% [3]. At the same time, some patients fear overkill and do not restrict their dietary intake, which in turn leads to excessive intake of potassium and phosphorus, which can lead to complications [4]. Therefore, healthcare professionals should strengthen the dietary guidelines for patients with MHD. On the one hand, they should strengthen patients' cognitive education about the importance of dietary management, and on the other hand, they can work together with a dietitian to develop a corresponding diet plan for patients according to their condition, weight, and blood pressure. The diet should conform to the principles of high calorie, low superior protein, low fat, low phosphorus, and low potassium as much as possible, prevent anaemia, ensure the intake and absorption of various nutrients, and actively prevent and treat malnutrition. Reasonable control of interdialytic weight gain (IDWG) during dialysis and keeping IDWG within the normal range are important measures to reduce complications, such as dialysis-associated hypotension, and reduce the morbidity and mortality rate of MHD patients, and patients' compliance with fluid intake is a key factor in the control of IDWG [5]. The patient's fluid intake compliance is a key factor in IDWG control [6]. Control of fluid intake is a problem for most MHD patients, and a significant proportion of MHD patients find controlling fluid intake the most difficult part of haemodialysis self-management because of severe thirst due to toxin retention in the body while limiting water intake [7]. Therefore, healthcare providers should give appropriate fluid intake instructions according to the patient's specific situation, explain the dangers of excessive fluid intake, teach patients techniques and methods to control fluid intake, self-monitor fluid intake, develop a fluid intake plan, and allow family members to monitor and control the patient's fluid intake.

The article "Application of a Computerized Decision Support System to Develop Care Strategies for Elderly Hemodialysis Patients" was published in 2021. Journal: J Healthc Eng.

Patients with MHD often suffer from varying degrees of mental health problems such as anxiety, depression, fear, stress, and even suicidal thoughts due to disease distress, frequent dialysis, impact of economic burden, and changes in social and family roles [8]. If psychological problems are not addressed promptly, they often affect the dialysis outcome and survival quality of patients and increase the risk of adverse events. Therefore, nursing staff should provide extended nursing interventions for patients' psychological problems, listen more to patients' emotional confessions, give humanistic care, and actively seek family and social support to enhance patients' confidence in treating the disease and improve their sense of well-being. They need to explore the problems in volume management of PD patients with poor adherence to volume management behaviours to improve the targeting of intervention programs and evaluate the impact of an IMCHB-based volume management intervention program on promoting volume management behaviours, improving volume balance, and improving quality of life in PD patients.

## 2. Related Work

With the aging of the global population, the increase in the number of elderly HD patients, prolongation of dialysis age, and special physiopathological conditions of the elderly, elderly HD patients are more prone to a variety of complications than other patients, and common complications include imbalance syndrome, heart failure, hypertension, diabetes, pruritus, and fractures [9]. A study by Shahmoradi et al. showed that the rate of arteriovenous access infections in elderly HD patients was as high as 37.5%, and the incidence of debilitation was 33.9% [10]. Palmer et al. found that 35.75% of elderly HD patients died of cardiovascular disease, 14.25% died of cerebrovascular disease, and 29% died of haemorrhagic disease, and the number of elderly patients who died of infection was significantly higher than that of young and middle-aged HD patients [11]. Moreover, given the special nature of the haemodialysis treatment form, ordinary elderly HD patients are mostly outpatients, and patients go home for convalescence after each haemodialysis. Therefore, elderly HD patients rely on themselves or their family members for various daily care [12]. The correctness and effectiveness of self-daily care for elderly HD patients cannot be measured, and healthcare professionals lack specific guidance tools to reasonably determine patients' care ability and thus cannot guide patients to effective care according to local conditions [13]. Self-management is the correct way of self-care, in which patients learn through health education, rely on their own ability to adopt effective behaviours to maintain or promote health, effectively monitor various complicating symptoms, detect them on time, and seek medical treatment on time.

The article "Application of a Computerized Decision Support System to Develop Care Strategies for Elderly Hemodialysis Patients" was published in 2021. Journal: J Healthc Eng.

Numerous scholars have achieved good results by intervening in patients through many different self-management approaches. Some scholars have shown that self-management can effectively correct patients' poor self-care habits, improve patients' alertness to changes in their disease, treatment compliance, and subjective motivation, thus reducing complications and improving patients' quality of survival [14]. The existing self-management scales for HD have deficiencies in diet, internal fistula care, and emotional communication. The contents of the scales are broad and pay little attention to the special physiological, psychological, cognitive, and safety problems of elderly HD patients. The existing self-management scales cannot truly reflect the problems in self-management of elderly HD patients. Therefore, it is necessary to develop a scientific and rigorous self-management scale to assess the self-management ability, deficits, and effects of elderly HD patients and provide evidence and direction for clinical care.

Niazkhani et al. used frequency domain analysis to extract pulse features [15]. Demiris et al. constructed a pulse recognition model using BP networks to improve the efficiency and accuracy of pulse diagnosis [16]. Regan constructed a pulse classification model by combining convolutional neural networks and recursive graphs, which further improved the efficiency and accuracy of pulse diagnosis [17]. Loftus et al. constructed a tongue classifier using vectorized neural networks and achieved very promising results [18]. In terms of health management, the development of smart mobile health and smart wearable devices has made it possible to collect health data from people's daily life. Health management is most closely connected to people and is especially important in the management of chronic diseases. Smart virtual nurses have emerged that can determine the basic state of a person based on the health data collected and can also remind patients of daily health management, such as medication, sleep, and exercise, providing all-around, whole-cycle health services.

## 3. Analysis of a Computerized Decision Support System to Develop Care Strategies for Elderly Hemodialysis Patients

### 3.1. Computerized Decision Support System Design

The heterogeneous clinical data analysis system designed in this paper needs to consider the heterogeneity and multimodality of clinical examination data, use deep learning as the main analysis technique, and combine with suitable fusion strategies to realize the fusion diagnosis of heterogeneous multimodal clinical data. For the implemented system, it should have flexible and scalable analysis methods to utilize as much information in as data as possible comprehensively to achieve more accurate diagnosis results. Moreover, since the system is mainly for the healthcare workers involved in clinical diagnosis, ease of use and robustness should be considered in the process of system implementation. In summary, the heterogeneous clinical data analysis system based on deep learning technology should have the following functions: before conducting analysis or training, the data should be preprocessed according to the data characteristics, which can provide a certain guarantee for the analysis or training effect [19]. Therefore, in the heterogeneous clinical analysis system, the corresponding data preprocessing module should be set according to the structure or mode of common clinical data, and the module should include the common preprocessing methods for this type of data, so that the preprocessing of the data can be easily completed using the processing methods in the system.

The article "Application of a Computerized Decision Support System to Develop Care Strategies for Elderly Hemodialysis Patients" was published in 2021. Journal: J Healthc Eng.

As one of the main functions of this system, when heterogeneous multimodal clinical data are input, the system should provide corresponding analysis means and fusion strategies to fuse and analyse the input data and output a comprehensive diagnosis conclusion of the disease. Considering the differences in diagnostic modalities of different diseases, multiple diagnostic models or fusion modalities can be considered for implementation to extend the application scenarios of the system. When the number of data structures or modalities generated by clinical diagnosis is not sufficient for fusion analysis, the system should have the ability to analyse single-modality clinical data. The unimodal clinical data analysis function should cover the common modalities in clinical data, such as electronic medical record text, medical images, and examination indicators. The analysis results should be visualized in the form of text, tables, or charts, and analysis reports should be formed for users to download.

According to the requirement analysis, the heterogeneous clinical data analysis system will be composed of four parts: front-end module, data preprocessing module, data analysis module, and data storage module. The front-end module realizes the interaction with users and mainly includes three functions: data preprocessing, data analysis, and result visualization and model download. The data preprocessing module provides preprocessing methods, such as word separation, format conversion, and data broadening for training or data to be analysed, while the data analysis module is responsible for calling the diagnostic model to make category judgment on the preprocessed data and return the diagnostic results. The data storage module of the system is mainly divided into file storage and database storage. File storage is to store the system model or user data that takes up more resources in the form of files; database storage uses a MySQL database to store user information, session logs, and other data. The general framework of the system is shown in Figure 1.

The article "Application of a Computerized Decision Support System to Develop Care Strategies for Elderly Hemodialysis Patients" was published in 2021. Journal: J Healthc Eng.

The front-end module is used to respond to user requirements and is mainly divided into four submodules: data preprocessing, unimodal clinical data analysis, heterogeneous multimodal clinical data analysis, and data download. The interface of each module is designed with the Element UI component library, and the MVVM model is used to realize the bidirectional data binding between the interface UI and the business model. This progressive framework enables responsive listening and dependency binding of components, and data interaction with functional modules through axis to complete page rendering. Users can upload and download data, analyse data, and set up models after entering the system through the login interface. The data expansion module can process the input data directly or receive data from the preprocessing module. The data enrichment function is implemented by calling the nibble library to convert the input image data into a multidimensional matrix, which is wrapped with functions for flipping, rotating, and transforming the matrix. The functions in the data augmentation module have no dependencies on each other, so they can be called in parallel, and the augmentation process outputs the same. The image data is also outputted after the augmentation process.

The main function of the data analysis module is to analyse the input clinical data and output prediction categories to provide an auxiliary diagnosis. To obtain more comprehensive information about the disease and improve the accuracy of prediction, the data analysis module fuses and analyses the heterogeneous multimodal data generated from the clinical diagnosis process. The data analysis module also includes a unimodal clinical data analysis function in consideration of the actual examination data that may have a more homogeneous structure or modality. The output of the module is divided into two types of classification categories and classification probabilities, and the return type can be selected by the front-end incoming parameters [20]. According to the fusion strategy designed and implemented in this paper, the heterogeneous multimodal clinical data fusion analysis submodule requires that the input data contain data from at least one modality in different structures, respectively. After reading the input data, the module recovers and calls the corresponding diagnostic models in the model library and obtains the model decision values. In the fusion method function, the decision values of each submodel are first stitched together, and the statistical calculation of the decision value arrays or matrices is performed using two fusion methods based on the decision-level fusion strategy.

The article "Application of a Computerized Decision Support System to Develop Care Strategies for Elderly Hemodialysis Patients" was published in 2021. Journal: J Healthc Eng.

This module is used to preprocess the input clinical data. Users can select the corresponding preprocessing module according to their needs, upload the data to be processed and configure the corresponding parameters, and save the data to the specified directory after the data preprocessing is completed. At present, the preprocessing process is mainly set up for image data and text data, which mainly includes the preprocessing process interface and parameter configuration for image data, including two functions of data augmentation and preprocessing. In the data expansion function, each expansion method generates the corresponding expanded data based on the original data and selecting multiple expansion methods means multiplying the original data. The preprocessing function includes data format conversion, spatial alignment, bias field correction, bone rejection, voxel normalization, resizing, and image cropping. Settings can be made to save data from each preprocessing step to a specified location or to keep only the final processed data.

### 3.2. Analysis of Nursing Strategy Methods for Elderly Hemodialysis Patients

Maintenance haemodialysis is one of the most important treatment modalities for ESRD patients. Its principle is to purify the blood by using the diffusion/convection function of the haemodialysis machine to remove various metabolic wastes, toxins, and excess electrolytes and water from the body to correct electrolyte disorders and acid-base homeostasis. The experiment is conducted to verify the operational reliability of the hybrid cloud fog computing-based architecture for integrating large health information resources. This experiment will use data redundancy rate, resource retrieval delay, and integration accuracy as experimental indexes, respectively. Among them, the data redundancy rate is calculated as follows:

(1) $$\begin{array}{c} S_{t}=\frac{A_{i}^{\prime }}{A}EW^{\prime }. \end{array}$$

The resource retrieval delay is calculated as follows:

(2) $$\begin{array}{c} Z_{c}=\frac{{\text{MIC}}^{\prime }}{A}P_{U}^{\prime }. \end{array}$$

The integration of the accuracy rate is calculated as follows:

(3) $$\begin{array}{c} Z_{z}=\frac{{\text{JA}}_{i}-{\text{MIC}}^{\prime }}{N}\text{ppd}. \end{array}$$

Accuracy (ACC) is the most common model evaluation criterion for classification tasks. It describes the number of samples correctly predicted by the model as a percentage of the total number of samples predicted and provides a good overview of the overall classification performance of the model. However, in scenarios where the classification task has category imbalance or is more concerned with positive sample segmentation, the accuracy rate is not a valid assessment of model performance. In this experiment, data augmentation was applied to the experimental dataset, which largely solved the category imbalance problem, but still focused more on the identification of the experimental positive samples (i.e., diseased patients) when evaluating the classification performance of the model, so the accuracy rate was only used as an index to judge whether the model training process was normal or not in this experiment and was not used to evaluate the final model performance.

The article "Application of a Computerized Decision Support System to Develop Care Strategies for Elderly Hemodialysis Patients" was published in 2021. Journal: J Healthc Eng.

In contrast to accuracy, which is a portrayal of the overall sample classification performance, precision is more concerned with the classification of positive samples. The accuracy rate describes the number of true positive samples as a percentage of the number of all samples predicted to be positive and represents how accurately the model predicts the correct outcome, which is calculated as shown in (4). Compared with the precision rate, the recall rate in (5) reflects the percentage of positive samples being successfully predicted among all predicted samples, so the recall rate is also known as the check-all rate.

(4) $$\begin{array}{c} \text{precision}=\frac{\text{TP}}{\text{TP}-\text{FP}}, \end{array}$$

(5) $$\begin{array}{c} \text{recall}=\frac{\text{TP}}{\text{TN}-\text{FN}}. \end{array}$$

Since this experiment classified subjects into three categories, AD, MCI, and CN, the classification task involved in the experiment was multicategorical. The definition of a positive sample for the autocategorisation task is that when calculating the assessment metric for each category, the category is considered as a positive sample alone and all other categories are considered as negative samples. Therefore, in the previously mentioned formula, TP represents the number of data with positive predicted value and positive true value among all the predicted samples; TN represents the number of data with negative predicted value and negative true value among all the predicted samples; FN represents the number of data with negative predicted value but positive true value among all the predicted samples; FP represents the number of data with positive predicted value and positive true value among all the predicted samples. Accordingly, FP represents the amount of data with positive predicted values but negative true values, as shown in Figure 2.

The article "Application of a Computerized Decision Support System to Develop Care Strategies for Elderly Hemodialysis Patients" was published in 2021. Journal: J Healthc Eng.

To ensure the model's ability to recognize positive samples while also focusing on the overall performance of the classification, the precision, recall, and ROC-AUC values of the model on the test samples are used as the comprehensive evaluation metrics of the model in the experiments. Since the experiments belong to the multiclassification task, it is necessary to use the multiclassification metric calculation method when calculating the evaluation metrics. The macroalgorithm, however, computes the precision rate of each class separately and then performs an arithmetic average with the formula (6), where precision is the precision rate of class I computed using formula (7). Macroalgorithm ignores the situation that the data of each class is not perfectly homogeneous and simply computes the metrics according to the number of classes, while, instead of multiplying the precision rate by a fixed number of categories as weights, the weighted algorithm multiplies the percentage of the category in the total sample size, as shown in (8), where *w*_*i*_ is the percentage of the category in the total sample size. Since the data volume of the three categories in the experimental data used in this paper is not exactly equal, the weighted algorithm is adopted for the calculation of the index.

(6) $$\begin{array}{c} {\text{precision}}_{\left(\text{micro}\right)}=\frac{\sum_{i=1}^{n}{\text{TP}}_{i}}{\sum_{i=1}^{n}{\text{TP}}_{i}-{\text{FP}}_{i}}, \end{array}$$

(7) $$\begin{array}{c} {\text{precision}}_{\left(\text{macro}\right)}=\sum_{i=1}^{n}{\text{precision}}_{i}*\frac{1}{n}, \end{array}$$

(8) $$\begin{array}{c} {\text{precision}}_{\left(\text{weighted}\right)}=\sum_{i=1}^{n}{\text{precision}}_{i}*w_{i}. \end{array}$$

The basic expert profile is described by the frequency and composition ratio. Expert positivity can be expressed by the expert positivity coefficient, that is, the return rate of valid correspondence questionnaires and the percentage of experts who gave corresponding opinions. Expert authority can be expressed by the expert authority coefficient (Cr), that is, the arithmetic mean of judgment coefficient (Ca) and familiarity coefficient (Cs). The mean, standard deviation, and other statistical indicators of importance and feasibility of modular indicators are used to express the degree of expert opinion coordination. Kendall's harmony coefficient and coefficient of variation (CV) are used to express the degree of expert opinion coordination. Standard deviation and other statistical indicators are used to indicate the degree of concentration of expert opinions. Kendall's harmony coefficient and coefficient of variation are used to indicate the degree of coordination of expert opinions.

The article "Application of a Computerized Decision Support System to Develop Care Strategies for Elderly Hemodialysis Patients" was published in 2021. Journal: J Healthc Eng.

The relationship between controllable factors and volume management behaviours led to the inspiration for constructing an intervention program: enhancing PD patients' knowledge and skills of volume control, including diet management and handling of daily volume overload problems, through group lectures or with the help of manuals; improving their ability to solve volume load problems and enhancing their sense of volume management self-efficacy. The level of hope influences patients' capacity management behaviour [21]. In the intervention, patients' belief in life can be enhanced by positive guidance from positive life experiences of patients and examples of pursuing dreams with illness. Themed activities such as “Enhancing Hope, Controlling Capacity” can be organized to enhance patients' beliefs about symptom control. In the interaction with patients, the positive perception of the meaning of dialysis treatment is promoted. For example, we will introduce the colourful dialysis life of kidney patients and make them realize that “dialysis is for a better life.” At the same time, patients are encouraged to participate in the interactive process of volume management to enhance their intrinsic sense of responsibility for disease management.

After building a medical corpus, the corpus can be used to construct a domain lexicon and to effectively split the medical texts to be analysed. The automatic construction process of its lexicon is shown in Figure 3.

Traditional text structuring or word separation methods generally only label information, such as lexical or sentence components, but lack attribute information, such as context for fixed phrases. Therefore, we need to break up the electronic medical record text into contents with XML tagging attributes and label them based on these contents, such as drug and disease names and other terms, for knowledge mining and analysis. Based on the dictionary, the identified words are labelled as different lexical properties, and new words (unregistered words) are identified among them by an improved algorithm, and the new words are recorded in the library and discovered by comparing them with the existing word list. Term recognition methods using N-Gram combined with various filtering rules can be used to identify new words in the corpus eventually, and the properties of each word are marked in XML. Based on the broken-up and structured electronic medical record text and information, such as sentence components and their corresponding contextual attributes, the semantic relationships between these contents are studied, and methods and models for analysing the semantic relationship network of these contents are proposed, which is the basic work for knowledge discovery.

The article "Application of a Computerized Decision Support System to Develop Care Strategies for Elderly Hemodialysis Patients" was published in 2021. Journal: J Healthc Eng.

In general hospital information systems, electronic medical records are stored in a semistructured form, and the basic information of patients (e.g., name, gender, ethnicity, etc.) exist in structured data tables, which are called structured data, and can be used directly in diagnosis and decision making and are not part of the content studied in this paper [22]. The subject of this paper is the narrative content of medical records written in natural language by physicians in electronic medical records, which are unstructured. Since many patients have complex causes or history of illness, it is difficult to describe such patient information completely in a structured storage structure, and natural language is often used to write treatment records in hospitals.

In the medical record dataset studied in this paper, each file is plain text data rather than semistructured data stored in a hospital information system. This means that in the case pages of an electronic medical record, structured data (e.g., information such as name, age, gender, etc.) and unstructured content (e.g., current medical history, history, personal history, etc.) are stored together and are difficult to distinguish. Therefore, we need to perform an initial splitting of these medical record files. The splitting requires processing the fields of the electronic medical record. The narrative text of ethology written by a physician inevitably has some grammatical problems in the form of expression, which generally do not affect the impact of the physician's judgment on the patient's condition. However, for computers, text with grammatical errors is an obstacle for automated programs to process. For example, in Chinese medical records, a comma in symbols is written as a comma. Therefore, for the subsequent computer to do standardized processing, it is necessary to replace the expression irregularities in the medical text to be processed beforehand.

## 4. Analysis of Results

### 4.1. System Performance Results

The size of the text dataset obtained from ADNI is small, and there is a great degree of category imbalance. Therefore, before training the model, the text data of electronic medical records are expanded by different orders of magnitude using the data augmentation module to increase the size of the dataset and balance the data categories at the same time.  Figure 4 shows the training accuracy of the TextCNN model with different dataset sizes. The 3*x* and 4*x* augmented datasets make the model fit slower but smoother, but finally, the augmented dataset achieves better accuracy than other datasets in the training. It can also be seen from Figure 4 that the scores of the evaluation metrics on the test set are proportional to the size of the dataset, which indicates that the model obtained better generalization after data augmentation, so the subsequent experiments were conducted on the text augmentation dataset.

The article "Application of a Computerized Decision Support System to Develop Care Strategies for Elderly Hemodialysis Patients" was published in 2021. Journal: J Healthc Eng.

The structured data for this experiment consisted of two data components. One part consists of data on the subject's demographic characteristics, medical history, and psychometric scores, and the other part is derived from the brain tissue volume data obtained by automated segmentation of the subject's MRI images. This processing step is based on the unsupervised segmentation method proposed by Leydig et al. The tissue of the brain MRI image is automatically segmented into 138 volumes of cortical and subcortical structures and segmented structures, and the volume data of the patient's brain tissue in the form of a data table is obtained by reading the segmentation report.  Figure 5 shows the partially segmented brain tissue and its volume data, with each column representing one brain tissue volume in 138 columns in cubic millimetres, and each row representing a different subject sample. The purpose of setting up the brain tissue volume data is to replace the laboratory indicator type data that were not available in the original experimental data for the experiment.

Since the two parts of the structured data were divided to generate different information at different stages of the diagnosis, the XGBoost algorithm was used to construct separate classifiers for the two parts of the structured data. In the classification model constructed for the structured data, such as basic subject information, medical history, and psychiatric examination, the objective function parameter was set to “multi:SoftMax” to return the predicted categories for the multiclassification task, and the metric was log loss for the multiclassification classification task. After parameter selection using grid search, the classification learning rate is set to 0.085 (default value is 0.3), and a smaller learning rate is found to have a better generalization effect by cross-validation. To prevent overfitting, the random sampling training sample ratio is set to 0.7 (default value is 1), which increases the randomness and makes the training robust to noise. In addition, the maximum depth of the tree is set to 3 (default value is 6) to reduce the complexity of the model.

The article "Application of a Computerized Decision Support System to Develop Care Strategies for Elderly Hemodialysis Patients" was published in 2021. Journal: J Healthc Eng.

It is used to measure the extent to which the content of the scale measures what the researcher wants to study. This is mainly reflected by measuring face validity and dimensional correlations, which are reflected in the correlation between the dimensions, correlation between the dimensions and the scale, and analysis by the scores of the dimensions and the total scale. The correlation coefficients of the entries in this study ranged from 0.27 to 0.72 for the total scale scores and from 0.59 to 0.72 for the dimensions concerning the total scale, as shown in Figure 6.

It consists of exploratory factor analysis and validation factor analysis. Usually, exploratory factor analysis can be used to discover the potential common factors of a scale and build a model based on a theory, and then, the validation factor analysis can be used to verify whether the model is consistent with the theoretical structure. In the present study, exploratory factor analysis was conducted to obtain a scale structure model with 25 items and five common factors based on a presurvey, and then, a validation factor analysis was applied to validate the existing scale structure model by a large sample of clinical survey.

After standardizing the duration of treatment across patients to the same time scale, more work is needed to discover medication characteristics based on the needs of the scenario, such as the duration of medication use in a particular patient group. The time–density reduction approach also has some negative effects, one issue being the distortion of absolute drug use, which means that the data processing cannot be used to calculate or compare absolute drug use across patients. In this case, we are still able to assess the relative importance of drugs in different modalities. In the previously mentioned example, the absolute number of days of drug D use for patient A is less than the absolute number of days for patient B, and patient A has a longer duration of use than patient B after the extension. This suggests that drug D plays a more important role in the treatment of patient A than in the treatment of patient B. Based on the desensitized data, we extracted the medication information from the electronic medical record text. In this process, we paid attention to both the duration and frequency of medication administration. The occurrence of drug names in a patient's treatment record was the format of frequency and duration. However, based on physician recommendations in this data experiment, we ignored the frequency of medications used during the day because the frequency is always related to the extent of disease and the dose of the medication, which is less important for clinical pathways and medication treatment planning. Therefore, for each patient, the processed electronic medical record data were in the form of a time-stamped medication list.

The article "Application of a Computerized Decision Support System to Develop Care Strategies for Elderly Hemodialysis Patients" was published in 2021. Journal: J Healthc Eng.

### 4.2. Results of Care Strategies for Hemodialysis Patients

The coefficients of variation of the importance of the indicators at all levels of the first round of expert consultation fluctuated from 0.00% to 20.94%, the coefficients of variation of feasibility fluctuated from 7.93% to 32.17%, and the Kendal coefficients of harmony fluctuated from 0.129 to 0.263. The coefficients of variation of the importance of indicators at all levels of the second round of expert consultation fluctuated from 0.00% to 21.22%, the coefficients of variation of feasibility fluctuated from 0.00% to 24.77%, and the coefficients of Kendal harmony fluctuated from 0.301 to 0.460.

The experts suggested that if the patients do not comply with the healthcare instructions and self-monitoring, there should be corresponding supervisory measures instead of simply providing some instructions to the patients. Therefore, combined with the expert's opinions and the discussion of the group, the following modifications were made. The platform can automatically detect whether patients view and learn health guidance, and if patients do not complete health guidance learning, the platform can remind patients to learn until they finish.

The report will be sent to the community healthcare, who will contact the patient or family for supervision. If the patient does not self-monitor on time, the patient will be reminded to upload. If the patient has not been recorded for a long time, the platform can report to the community healthcare, and the community healthcare will supervise. When patients view and study medical guidance on time, regularly conduct health self-assessment, self-monitor daily on time, and read health information, kidney circle release news, and so on, they can get the corresponding points reward, monthly for the top patients to give encouragement, or certain material rewards, to enhance the user's enthusiasm and user stickiness to use the extended care information platform. Some experts suggest that the exercise situation of patients should be evaluated regularly. Targeted exercise guidance should be provided according to the exercise situation of patients, so the “A2-7 exercise evaluation” can be added. The exercise situation of patients can be evaluated regularly by combining subjective and objective methods. The corresponding exercise prescriptions can be formulated for patients according to the evaluation results, as shown in Figure 7. Based on the assessment results, the corresponding exercise prescriptions will be formulated for patients, as shown in Figure 8.

The article "Application of a Computerized Decision Support System to Develop Care Strategies for Elderly Hemodialysis Patients" was published in 2021. Journal: J Healthc Eng.

Analysing Figure 8, compared with traditional method 1 and traditional method 2, the acceleration ratio and parallel efficiency of the method in this paper are higher. In case of increasing the number of cores, traditional method 1 computation time increases instead, leading to a significant reduction in overall parallel efficiency, which is mainly because traditional method 1 does not chunk the health data stream, leading to an increase in communication overhead. When traditional method 2 is used, although the computation time decreases to a certain extent and the acceleration ratio increases to a certain extent when the number of cores increases, the reduction in parallel efficiency is significantly better than that of traditional method 1, and the overall computation performance is significantly inferior to that of this paper. Using this paper's method can greatly reduce the parallel computation time while achieving a good acceleration ratio and parallel efficiency, and the parallel computation time is significantly reduced when the number of cores increases, mainly because this paper's method processes the health data stream in chunks, reduces the data scale and condition number, enhances data convergence, reduces the communication overhead, enhances the overall parallel computation efficiency, and has superior computational performance.

## 5. Conclusion

Given the disease factors and the special nature of dialysis treatment, maintenance haemodialysis often faces various physiological or psychological problems, and comprehensive and accurate extended care services are significant for prolonging patients' survival, improving their prognosis, and enhancing their self-management ability and quality of life. In this study, we constructed the content of a mobile healthcare-based information platform for extended care of maintenance haemodialysis patients through extensive literature reading, qualitative interviews, and expert correspondence method and explored how to provide intelligent extended care services for maintenance haemodialysis patients by using mobile healthcare information technology and combining the hospital–community–home integrated extended care model. This study finalized the module content system of the mobile medical-based extended care information platform for maintenance haemodialysis patients through the expert consultation method, which contains three primary indicators, 18 secondary indicators, and 82 tertiary indicators. The experts consulted had high professional representativeness and authority, they were well-motivated, and their opinions were coordinated and concentrated. The module content, thus constructed, was scientific and reliable, which provided a basis for the next development of the information platform and the promotion of the R&D results.

The article "Application of a Computerized Decision Support System to Develop Care Strategies for Elderly Hemodialysis Patients" was published in 2021. Journal: J Healthc Eng.

## Figures and Tables

**Figure 1:** Computerized decision support system.

**Figure 2:** Framework of nursing strategy approach.

**Figure 3:** Automatic policy construction process.

**Figure 4:** Training accuracy of different sized datasets.

**Figure 5:** Volume data.

**Figure 6:** Correlation coefficient between the scores of each item and the total score of the scale.

**Figure 7:** Degree of coordination.

**Figure 8:** Load balancing response spectrum.

## Data Availability

Data sharing is not applicable to this article as no datasets were generated or analysed during the current study.
